The article "TiO2 NPs/h-BN: Preparation and catalytic activities of a novel AP catalyst" was published in 2022. Journal: Front Chem.

# TiO_2_ NPs/h-BN: Preparation and catalytic activities of a novel AP catalyst

**DOI:** 10.3389/fchem.2022.947052

**Published:** 2022-07-22

**Authors:** Jun Zhao, Nengmei Deng

**Affiliations:** West Anhui University, Lu’an, China

**Keywords:** TiO_2_ NPs/h-BN, AP, BN, thermal decomposition, catalytic

## Abstract

The thermal decomposition performance of an oxidizer directly determines the thrust and specific impulse properties of the solid propellant. Hexagonal boron nitride (h-BN) has the characteristics of high catalytic activity and good stability, which can improve the heat release and decomposition temperature of the oxidant, and then improve the energy performance of the propellant. In this study, a novel hybrid material TiO_2_ NPs/h-BN was successfully prepared by *in situ* growth, and it was found that when 5 wt.% TiO_2_ NPs/h-BN was added, the initial decomposition temperature of ammonium perchlorate (AP) decreased by 67.6°C. Due to the addition of TiO_2_, the gap between the h-BN layers as well as the specific surface increased, which optimized its thermocatalytic performance, and it also proposed a catalytic mechanism for the thermal decomposition process of AP.

## Introduction

Solid propellants consisted of oxidants, binders, metal burners, and other additional components. Among them, the oxidant, as the source of oxygen required for propellant combustion, occupied more than 70% of the propellant, and its thermal decomposition performance had a great influence on the combustion of the propellant. Among these oxidants, AP had the advantages of high effective oxygen content and high density and was one of the most commonly used oxidants in solid propellants (Li et al., 2021). However, the properties of AP, such as high thermal decomposition temperature, high reaction activation energy, low heat release, and non-concentrated heat release, were important factors restricting the development of high-energy solid propellants (Huang et al., 2021). Therefore, in order to meet the needs of modern aerospace technology and the world arms race for high-energy solid propellants, it is necessary to improve the thermal decomposition performance of AP (Li et al., 2020a).

Recently, two-dimensional atomic crystals are now attracting increasing attention in various fields and applications, inspired by the “graphene gold rush” (Sun et al., 2018; Li et al., 2020b; Shen et al., 2021a; Shen et al., 2021b; Li et al., 2022). As a typical graphene-like material, h-BN has attracted great research interest because of its good oxidation resistance up to 850°C, excellent acid chemical stability, high thermal conductivity, excellent elastic modulus, and good mechanical flexibility (Sun et al., 2016). More importantly, h-BN has been identified as a promising dielectric layer or protective encapsulation material (Li et al., 2012; Shen et al., 2020; Wang et al., 2020). Metal oxide semiconductor materials had the advantages of heat resistance, antitoxicity, photosensitivity, heat sensitivity, and impurity sensitivity and were suitable for modulation, so they have attracted much attention in the field of catalysis (Thomas et al., 2016; Zhu et al., 2016; Li et al., 2017; Li et al., 2020c). Therefore, we propose a technical scheme for the preparation of novel composite catalysts using few-layer boron nitride–supported TiO_2_ (Medvecká et al., 2018).

The article "TiO2 NPs/h-BN: Preparation and catalytic activities of a novel AP catalyst" was published in 2022. Journal: Front Chem.

In this work, we first used a purely physical green peeling method—liquid nitrogen impact method to peel off the multilayer boron nitride (BN)—and then used a one-step synthesis *in situ* growth method to obtain the target product TiO_2_ NPs/h-BN, and the thermal catalytic effect of the composite on AP was studied. The results showed that the decomposition temperature of ammonium perchlorate decreased by 67.6°C when 5% (mass fraction) was added. Also, the catalytic mechanism was studied.

## Experimental

### Chemicals and apparatus

Ammonium chloride (99%), aluminite powder (99.99%), BBr_3_ (AR), hydrochloric acid (35%), ethanol, glacial acetic acid, butyl titanate, and AP (AR) were obtained from Aladdin (Shanghai, China).

### Preparation of h-BN

Synthesis experiments were performed in a N_2_-flow glove box. NH_4_Cl (0.150 mol), Al (0.100 mol), and BBr_3_ (0.050 mol) were put into a stainless steel autoclave with a volume of 50 ml. The autoclave was sealed and heated in an oven at a ramp rate of 10°C/min from room temperature to 500°C and held at 500°C for 10 h (Huang et al., 2018). The product was dried under vacuum at 80°C for 10 h.

### Preparation of h-BNNS

The prepared 5 g of white powder was weighed, placed in a crucible, placed in a muffle furnace, heated to 800°C at a heating rate of 10°C, and kept warm for 30 min. At the end of heat preservation, it was quickly taken out, poured into the prepared liquid nitrogen (L-N_2_) until the L-N_2_ gasified completely. The white powder was suddenly cooled, liquid nitrogen was rapidly evaporated, and the steam-impinging boron nitride powder was boiled. The essence of this strategy lies in the combination of a high temperature–triggered expansion of bulk h-BN and a subsequent L-N_2_ gasification that exfoliates the h-BN (Li et al., 2019). Repeat the aforementioned steps three times to obtain the target product (h-BNNS). Scheme 1A was gas exfoliation of h-BN triggered by thermal expansion, and Scheme 1B was the photograph of TiO_2_ NPs/h-BN.

The article "TiO2 NPs/h-BN: Preparation and catalytic activities of a novel AP catalyst" was published in 2022. Journal: Front Chem.

**SCHEME 1:** **(A)** Gas exfoliation of h-BN triggered by thermal expansion. **(B)** Photograph of TiO_2_ NPs/h-BN.

### Preparation of TiO_2_ NPs/h-BN

A volume of 5.0 ml ethanol and 2.0 ml of glacial acetic acid were placed in a beaker, then 6.8 ml of butyl titanate was added to it, and at 30°C, under magnetic stirring for 10 min, 0.8 g of h-BNNS was added and labeled as Solution A (Li et al., 2018). Into another beaker was added 4.0 ml of deionized water, 5.0 ml of ethanol, and 7.2 ml of glacial acetic acid and magnetically stirred for 10 min to uniformly mix to obtain Solution B (Xue et al., 2011). After the dropwise addition was completed, stirring was continued for 20 min to obtain a uniform solution. It was allowed to stand at room temperature for 24 h to form a gel and dried in a drying oven at 80°C for 12 h. The ground samples were placed in a muffle furnace, calcined at 400°C for 2 h, and then cooled naturally to obtain TiO_2_ NPs/h-BN.

## Results and discussion

### Sample characterization

The FT-IR result is shown in Figure 1A. The two absorption peaks at 1388.6 cm^−1^ and 813.4 cm^−1^ are the in-plane stretching vibration of B-N and the out-of-plane bending B-N-B vibration, respectively. The absorption peak at 3433.8 cm^−1^ is the in-plane stretching vibration of N-H (Thomas et al., 2008). The Raman spectrum showed that the G-band frequency of h-BNNS was shifted up relative to that of bulk h-BN (1366.8 cm^−1^ vs. 1365.8 cm^−1^; Figure 1B). The G-band shift could be attributed to the reduction of h-BN layers, which led to higher in-plane strain and weaker interlayer interactions.

**FIGURE 1:** **(A)** FT-IR spectra of h-BN. **(B)** Raman characterizations of bulk h-BN and h-BNNS.

As shown in Figure 2, the scanning electron microscope images of the parent h-BN and h-BNNS are shown in Figures 2A,B. Compared with the bulky h-BN precursors, h-BNNS was much smaller in size and possessed nanosheet-like morphology (Lei et al., 2018).

**FIGURE 2:** Characterization of exfoliated h-BNNS. **(A)** SEM of h-BN. **(B)** SEM of h-BNNS.

The SEM results also proved that we successfully prepared TiO_2_ NPs/h-BN, as shown in Figure 3. TiO_2_ NPs were uniformly dispersed on the surface of the h-BN (Hosseini et al., 2018). In addition, EDS showed that TiO_2_ was uniformly distributed on boron nitride nanoparticles.

**FIGURE 3:** SEM of TiO_2_ NPs/h-BN **(A,B)** and EDS of TiO_2_ NPs/h-BN **(C–E)**.

Figure 4 shows the TEM of TiO_2_ NPs/h-BN. We found that TiO_2_ had microspherical morphology, and the outer layer was covered by h-BN. It was consistent with the SEM characterization results.

**FIGURE 4:** TEM of TiO_2_ NPs/h-BN

Figure 5A shows the XPS of TiO_2_ NPs/h-BN. The characteristic peaks at 458.9 and 464.7 eV correspond to the binding energies of Ti 2p1/2 and Ti 2p3/2, respectively, indicating that Ti was at positive 4 valence, Ti^4+^. Nitrogen adsorption/desorption isotherms were conducted at 77 K to study the textural properties of TiO_2_ NPs/h-BN (Figure 5B). Because of its spherical structure, its specific surface area was large. Based on the nitrogen adsorption and desorption curves, the BET surface areas of TiO_2_ NPs/h-BN was 112.5 m^2^ g^−1^.

The article "TiO2 NPs/h-BN: Preparation and catalytic activities of a novel AP catalyst" was published in 2022. Journal: Front Chem.

**FIGURE 5:** **(A)** XPS of TiO_2_ NPs/h-BN. **(B)** N2 adsorption/desorption isotherms of TiO_2_ NPs/h-BN.

### Catalytic activities of TiO_2_ NPs/h-BN in the thermal decomposition of AP

In order to fully demonstrate the effectiveness of TiO_2_ NPs/h-BN in catalyzing the thermal decomposition of AP, we carried out research work by means of thermal analysis. As shown in Figure 6A, compared with the DTA curve of pure AP, the decomposition peak temperature of AP was advanced to 395.7°C by the catalysis of TiO_2_. After the addition of TiO_2_ NPs/h-BN, the HTD temperature was further advanced to 380.8°C, confirming the intrinsic catalytic effect of TiO_2_ NPs/h-BN on AP. This conclusion is also confirmed by the TGA-DTG results, as shown in Figure 5B; in the TGA curve of AP, the two characteristic weight loss steps correspond to the LTD and HTD phases where the weight loss rate reaches 25% and 74%, respectively (Jacobs and Russell-Jones, 1968; Morales- Verdejo et al., 2018; Yuan et al., 2018).

**FIGURE 6:** **(A)** DTA curves of pure AP; AP mixed with TiO_2_ (5%); and AP mixed with TiO_2_ NPs/h-BN (5%). **(B)** TG/DTG curves of AP mixed with TiO_2_ NPs/h-BN (5%).

As shown in Figure 7, we collected samples before and after thermal catalysis and performed by XRD. Diffraction peaks existed in all samples: 2θ = 25.5°, 37.8°, 48.2°, 53.7°, 55.2°, 62.6°, 68.9°, 70.4°, and 75.3°, which corresponding to this diffraction peak was (0002), (004), (112), (200), (0004), (204), (116), (220), and (215); these diffraction peaks were compared with h-NB and TiO_2_. We collected the catalytic effect and recovery rate of the TiO_2_ NPs/h-BN after two cycles of thermocatalysis in Table 1.

**FIGURE 7:** XRD of TiO_2_ NPs/h-BN before and after thermal catalysis.

**TABLE 1:** Recycling and stability of TiO_2_ NPs/h-BN.

Cycle	Recovery rate	Decomposition temperature of AP (°C)
1	98 (%)	380.8
2	95 (%)	380.3
3	92 (%)	380.7

### Catalytic mechanisms

The addition of h-BNNS inhibited the agglomeration of TiO_2_ particles during the preparation process and synergistically enhanced the catalytic activity by forming a hybrid structure (Al- Ani and Hogarth, 1985; Al- Kuhaili et al., 2002; Cui et al., 2012; Xu et al., 2013; Zhao et al., 2016). The catalytic effect of h-BN was attributed to the negatively charged h-BN surface (Shen et al., 2006; Tu et al., 2014), which facilitated the transfer of induced holes to the TiO_2_ surface due to the electrostatic attraction between them to form OH^−^ or **·**OH radicals, which initiated subsequent surface degradation reaction (Li et al., 2008; Sharma et al., 2014; Eslami et al., 2017).

The article "TiO2 NPs/h-BN: Preparation and catalytic activities of a novel AP catalyst" was published in 2022. Journal: Front Chem.

The catalytic process is shown in Figure 8. The adsorption of HClO_4_ and NH_3_ obtained from the first decomposition prevented the decomposition of AP. (Reid et al., 2007; Li et al., 2015a; Li et al., 2015b; Abazari and Mahjoub, 2017). As the temperature increased, conduction band electrons and valence band holes were generated on the surface of h-BN, and the generated electrons reacted with HClO_4_, resulting in the reduction of HClO_4_ to a superoxide radical anion. O_2_^−^ further reacted with NH_3_ to generate H_2_O, NO_2_, and N_2_O (Zhang et al., 2014; Jain et al., 2019).

**FIGURE 8:** Schematic of the thermal decomposition of AP with TiO_2_ NPs/h-BN as additives; CB, conduction band; VB, valence band.

## Conclusion

A novel TiO_2_ NPs/h-BN hybrid material with strong interfacial interactions has been successfully constructed by *in situ* solvothermal growth. Experiments showed that the TiO_2_ NPs/h-BN exhibited a good catalytic effect on the decomposition of AP, which reduced the high thermal decomposition temperature of AP by 67.6°C. At the same time, we deeply analyzed TiO_2_ NPs/h-BN as a novel catalyst to provide a mechanism for thermal decomposition of AP.

## Data Availability

The original contributions presented in the study are included in the article/Supplementary Material; further inquiries can be directed to the corresponding author.

## References

[B1] AbazariR.MahjoubA. R. (2017). Potential applications of magnetic β-AgVO3/ZnFe2O4 nanocomposites in dyes, photocatalytic degradation, and catalytic thermal decomposition of ammonium perchlorate. Ind. Eng. Chem. Res. 56, 623–634. 10.1021/acs.iecr.6b03727

[B2] Al-AniS. K. J.HogarthC. A. (1985). Int.A study of optical absorption in tellurite and tungsten-tellurite glasses. J. Electron. 58, 123

[B3] Al-KuhailiM. F.DurraniS. M. A.KhawajaE. E.ShirokoffJ. (2002). Effects of preparation conditions on the optical properties of thin films of tellurium oxide. J. Phys. D. Appl. Phys. 35, 312–915. 10.1088/0022-3727/35/9/312

[B4] CuiX. Q.ZhaoY. H.ChuY. Q. (2012). The large sky area multi-object fiber spectroscopic telescope (LAMOST). Res. Astronomy Astrophysics 12, 1197. 10.1117/12.319250

[B5] EslamiA.JuibariN. M.HosseiniS. G.AbbasiM. (2017). Synthesis and Characterization of CuO nanoparticles by the chemical liquid deposition method and investigation of its catalytic effect on the thermal decomposition of ammonium perchlorate. Cent. Eur. J. Energy Mat. 14, 152–168. 10.22211/cejem/67560

The article "TiO2 NPs/h-BN: Preparation and catalytic activities of a novel AP catalyst" was published in 2022. Journal: Front Chem.

[B6] HosseiniS. G.ZareiM. A.TolotiS. J. H.KardanH.AlaviM. A. (2018). A facile synthesis of boron nanostructures and investigation of their catalytic activity for thermal decomposition of ammonium perchlorate particles. J. Therm. Anal. Calorim. 131, 925–935. 10.1007/s10973-017-6595-7

[B7] HuangT.HaoW. J.JinB.ZhangJ. H.GuoJ. K.LuoL. Q. (2021). Novel energetic coordination compound [Cu (AT) _4_] Cl_2_ for catalytic thermal decomposition of ammonium perchlorate. J. Solid State Chem. 304, 122622. 10.1016/j.jssc.2021.122622

[B8] HuangY.ChenD.HuX.QianY.LiD. (2018). Synthesis and characterization of “ravine-like” BCN compounds with high capacitance. Materials 8, 209. 10.3390/ma11020209 PMC584890629382167

[B9] JacobsP. W. M.Russell-JonesA. (1968). Sublimation of ammonium perchlorate. J. Phys. Chem. 72, 202–207. 10.1021/j100847a038

[B10] JainS.KhireV. H.KandasubramanianB. (2019). Barium titanate: a novel perovskite oxide burning rate modifier for HTPB/AP/Al based composite propellant formulations. Pune: Propellants, Explosives, Pyrotechnics.

[B11] LeiL.KongT.ZhuP.KangZ.TianX.WangL. (2018). Self-assembly of TiO_2_ nanofiber-based microcapsules by spontaneously evolved multiple emulsions. Langmuir 34, 8785–8791. 10.1021/acs.langmuir.8b01472 29983067

[B12] LiH.WuC.LiY.ZhangJ. (2012). Superior activity of MnOx-CeO_2_/TiO_2_ catalyst for catalytic oxidation of elemental mercury at low flue gas temperatures. Appl. Catal. B Environ. 111, 381–388. 10.1016/j.apcatb.2011.10.021

[B13] LiK.LeiY.LiaoJ.ZhangY. (2021). Facile synthesis of MXene-supported copper oxide nanocomposites for catalyzing the decomposition of ammonium perchlorate. Inorg. Chem. Front. 8, 1747–1761. 10.1039/d0qi01337d

[B14] LiK.WangB.BolatibiekeD.NanD. H.LiQ. (2020). Pyrolysis of biomass impregnated with ammonium dihydrogen phosphate for polygeneration of phenol and supercapacitor electrode material. Front. Chem. 8, 436. 10.3389/fchem.2020.00436 32509737PMC7248177

[B15] LiL.SunX.QiuX.XuJ.LiG. (2008). Nature of catalytic activities of CoO nanocrystals in thermal decomposition of ammonium perchlorate. Inorg. Chem. 47, 8839–8846. 10.1021/ic8008283 18763761

[B16] LiQ.HeY.PengR. (2015). Graphitic carbon nitride (g-C_3_N_4_) as a metal-free catalyst for thermal decomposition of ammonium perchlorate. RSC Adv. 5, 24507–24512. 10.1039/c5ra01157d

[B17] LiQ.HeY.PengR. (2015). One-step synthesis of SnO_2_ nanoparticles-loaded graphitic carbon nitride and their application in thermal decomposition of ammonium perchlorate. Eur. J. Inorg. Chem. 24, 4062–4067. 10.1002/ejic.201500507

The article "TiO2 NPs/h-BN: Preparation and catalytic activities of a novel AP catalyst" was published in 2022. Journal: Front Chem.

[B18] LiS. J.ChenJ. L.HuS. W.WangH. L.ChenX. B. (2020). Facile construction of novel Bi_2_WO_6_/Ta_3_N_5_ Z-scheme heterojunction nanofibers for efficient degradation of harmful pharmaceutical pollutants. Chem. Eng. J. 402, 126165. 10.1016/j.cej.2020.126165

[B19] LiS. J.HuS. W.JiangW.ZhangJ. L.XuK. X.WangZ. H. (2019). *In situ* construction of WO_3_ nanoparticles decorated Bi_2_MoO_6_ microspheres for boosting photocatalytic degradation of refractory pollutants. J. colloid interface Sci. 556, 335–344. 10.1016/j.jcis.2019.08.077 31465964

[B20] LiS. J.HuS. W.JiangW.ZhouY. T.LiuJ. S.WangZ. H. (2018). Facile synthesis of cerium oxide nanoparticles decorated flower-like bismuth molybdate for enhanced photocatalytic activity toward organic pollutant degradation. J. colloid interface Sci. 530, 171–178. 10.1016/j.jcis.2018.06.084 29982008

[B21] LiS. J.ShenX. F.LiuJ. S.ZhangL. S. (2017). Synthesis of Ta_3_N_5_/Bi_2_MoO_6_ core-shell fiber-shaped heterojunctions as efficient and easily recyclable photocatalysts. Environ. Sci. Nano 4, 1155–1167. 10.1039/c6en00706f

[B22] LiS. J.WangC. C.ChenJ. L.ZhangP.LiX.ChenX. B. (2022). Facile fabrication of TaON/Bi2MoO6 core–shell S-scheme heterojunction nanofibers for boosting visible-light catalytic levofloxacin degradation and Cr (VI) reduction. Chem. Eng. J. 428, 131158. 10.1016/j.cej.2021.131158

[B23] LiS. J.WangC. C.LiuY. P.XueB.ChenJ. L.WangH. W. (2020). Facile preparation of a novel Bi_2_WO_6_/calcined mussel shell composite photocatalyst with enhanced photocatalytic performance. Catalysts 10, 1166. 10.3390/catal10101166

[B24] MedveckáV.KováčikD.ZahoranováA.ČernákM. (2018). Atmospheric pressure plasma assisted calcination by the preparation of TiO_2_ fibers in submicron scale. Appl. Surf. Sci. 428, 609–615. 10.1016/j.apsusc.2017.09.178

[B25] Morales-VerdejoC.CamaradaM. B.ArroyoJ. L.PoveaP.CarreñoG.ManriquezJ. M. (2018). Effect of the homo- and heterobimetallic compounds derived from s-indacene on the thermal decomposition of ammonium perchlorate. J. Therm. Anal. Calorim. 131, 353–361. 10.1007/s10973-017-6534-7

[B26] ReidD. L.RussoA. E.CarroR. V.StephensM. A.LePageA. R.SpaldingT. C. (2007). Nanoscale additives tailor energetic materials. Nano Lett. 7, 2157–2161. 10.1021/nl0625372

[B27] SharmaJ. K.SrivastavaP.SinghG. (2014). Nanocatalysts: Potential burning rate modifier for composite solid propellants. Mat. focus 3, 81–91. 10.1166/mat.2014.1154

[B28] ShenG.ChenD.LeeC. J. (2006). Hierarchical saw-like ZnO nanobelt/ZnS nanowire heterostructures induced by polar surfaces. J. Phys. Chem. B 110, 15689–15693. 10.1021/jp0630119 16898712

The article "TiO2 NPs/h-BN: Preparation and catalytic activities of a novel AP catalyst" was published in 2022. Journal: Front Chem.

[B29] ShenX. F.YangJ. Y.ZhengT.WangQ.ZhuangH. F.ZhengR. N. (2020). Plasmonic pn heterojunction of Ag/Ag_2_S/Ag_2_MoO_4_ with enhanced vis-NIR photocatalytic activity for purifying wastewater. Sep. Purif. Technol. 251, 117347. 10.1016/j.seppur.2020.117347

[B31] ShenX. F.ZhangY.ShiZ.ShanS. D.LiuJ. S.ZhangL. S. (2021a). Construction of C_3_N_4_/CdS nanojunctions on carbon fiber cloth as a filter-membrane-shaped photocatalyst for degrading flowing wastewater. J. Alloys Compd. 851, 156743. 10.1016/j.jallcom.2020.156743

[B30] ShenX. F.YanZ.SongB. B. T.ChenF.XueQ. Q.ShanS. D. (2021b). Magnetically recyclable and remarkably efficient visible-light-driven photocatalytic hexavalent chromium removal based on plasmonic biochar/bismuth/ferroferric oxide heterojunction. J. Colloid Interface Sci. 590, 424–435. 10.1016/j.jcis.2021.01.095 33561592

[B32] SunJ.LuC.SongY.JiQ.SongX.LiQ. (2018). Recent progress in the tailored growth of two-dimensional hexagonal boron nitride via chemical vapour deposition. Su zhou: Chemical Society Reviews. 10.1039/c8cs00167g29717732

[B33] SunW.MengY.FuQ.WangF.WangG.GaoW. (2016). High-yield production of boron nitride nanosheets and its uses as a catalyst support for hydrogenation of nitroaromatics. ACS Appl. Mat. Interfaces 8, 9881–9888. 10.1021/acsami.6b01008 27023711

[B34] ThomasA.FischerA.GoettmannF.AntoniettiM.MüllerJ. O.SchlöglR. (2008). Graphitic carbon nitride materials: variation of structure and morphology and their use as metal-free catalysts. J. Mat. Chem. 18, 4893. 10.1039/b800274f

[B35] ThomasJ. C.DemkoA. R.TE.ReidD. L.SealS.PetersenE. L. (2016). Mechanical properties of composite AP/HTPB propellants containing novel titania nanoparticles. Prop. Explos. Pyrotech. 41, 822–834. 10.1002/prep.201600090

[B36] TuD.XuC. N.FujioY.KamimuraS.SakataY.UenoN. (2014). Phosphorescence quenching by mechanical stimulus in CaZnOS: Cu. Appl. Phys. Lett. 105, 011908. 10.1063/1.4890112

[B37] WangX.HuW.HuY. (2020). Polydopamine-bridged synthesis of ternary h-BN@ PDA@ TiO_2_ as nanoenhancers for thermal conductivity and flame retardant of polyvinyl alcohol. Front. Chem. 8, 587474. 10.3389/fchem.2020.587474 33134281PMC7552804

[B38] XuJ.ZhangL.ShiR.ZhuY. (2013). Chemical exfoliation of graphitic carbon nitride for efficient heterogeneous photocatalysis. J. Mat. Chem. A Mat. 1, 14766. 10.1039/c3ta13188b

[B39] XueJ.Sanchez-YamagishiJ.BulmashD.JacquodP.DeshpandeA.WatanabeK. (2011). Scanning tunnelling microscopy and spectroscopy of ultra-flat graphene on hexagonal boron nitride. Nat. Mat. 10, 282–285. 10.1038/nmat2968 21317900

[B40] YuanY. J.YangY.LiZ.ChenD.WuS.FangG. (2018). Promoting charge separation in g-C_3_N_4_/graphene/MoS_2_ photocatalysts by two-dimensional nanojunction for enhanced photocatalytic H_2_ production. ACS Appl. Energy Mat. 1, 1400–1407. 10.1021/acsaem.8b00030

The article "TiO2 NPs/h-BN: Preparation and catalytic activities of a novel AP catalyst" was published in 2022. Journal: Front Chem.

[B41] ZhangJ.ZhangM.YangC.WangX. (2014). Nanospherical carbon nitride frameworks with sharp edges accelerating charge collection and separation at a soft photocatalytic interface. Adv. Mat. 26, 4121–4126. 10.1002/adma.201400573 24706532

[B42] ZhaoJ.JinB.PengR.LiuQ.TanB.ChuS. (2016). Synthesis and characterization of a new energetic salt 1H-pyrazole-1-carboxamidine dinitramide and its thermal properties. J. Therm. Anal. Calorim. 124, 1431–1439. 10.1007/s10973-016-5315-z

[B43] ZhuW.GaoX.LiQ.LiH.ChaoY.LiM. (2016). Controlled gas exfoliation of boron nitride into few-layered nanosheets. Angew. Chem. Int. Ed. Engl. 55, 10924–10928. 10.1002/ange.201605515 27444210

